# Multidisciplinary management for Peutz–Jeghers syndrome and prevention of vertical transmission to offspring using preimplantation genetic testing

This article has been retracted.

**DOI:** 10.1186/s13023-022-02221-z

**Published:** 2022-02-21

**Authors:** Xiqiao Xu, Ruifeng Song, Kaiyue Hu, Ya Li, Haixia Jin, Bing Chen, Wenyan Song, Yile Zhang, Jiawei Xu, Yingpu Sun

**Affiliations:** 1 Center for Reproductive Medicine, Henan Key Laboratory of Reproduction and Genetics, The First Affiliated Hospital of Zhengzhou University, Zhengzhou, 450052 Henan China; 2 Henan Key Laboratory of Reproduction and Genetics, The First Affiliated Hospital of Zhengzhou University, Zhengzhou, China; 3 Henan Provincial Obstetrical and Gynecological Diseases (Reproductive Medicine) Clinical Research Center, The First Affiliated Hospital of Zhengzhou University, Zhengzhou, China; 4 Henan Engineering Laboratory of Preimplantation Genetic Diagnosis and Screening, The First Affiliated Hospital of Zhengzhou University, Zhengzhou, China; 5 Department of Gastroenterology, First Affiliated Hospital of Zhengzhou University, Zhengzhou, China

**Keywords:** Rare diseases, Peutz–Jeghers syndrome (PJS), Preimplantation genetic testing for monogenic defects (PGT-M), Multi-disciplinary team (MDT), *STK11*

## Abstract

**Background:**

Peutz Jeghers syndrome (PJS) is an autosomal dominant genetic disorder caused by STK11 mutation with a predisposition to gastrointestinal polyposis and cancer. PJS patients suffer poor quality of life and are highly concerned about whether deleterious mutations transmit to their offspring. Therefore, this study aimed to propose feasible clinical management and provide effective preimplantation genetic testing for monogenic defect (PGT-M) strategies to protect offspring from inheriting the disease.

**Methods:**

A hospital-based clinical retrospective analysis reviewing the clinical characteristics and fertility aspects was first conducted on 51 PJS patients at the First Affiliated Hospital of Zhengzhou University between January 2016 and March 2021. Among the 51 patients, the PGT-M strategy was further carried out in 4 couples, which started with a biopsy of the trophectoderm cells of embryos and whole genome amplification using multiple displacement amplification. Thereafter, single nucleotide polymorphism linkage analyses based on karyomapping were performed with copy number variations of the embryos identified simultaneously. Finally, prenatal diagnosis was used to verify the validity of the PGT-M results.

**Results:**

A comprehensive management flowchart adopted by the multidisciplinary team model was formulated mainly focusing on clinical genetic and gastrointestinal aspects. Under the guidelines of this management, 32 embryos from 4 PJS pedigrees were diagnosed and 2 couples successfully conceived healthy babies free of the *STK11* pathogenic mutation.

**Conclusions:**

Our comprehensive management could help affected families avoid having children with PJS through preimplantation genetic testing and provide meaningful guidance for multidisciplinary clinical practice on PJS.

**Supplementary Information:**

The online version contains supplementary material available at 10.1186/s13023-022-02221-z.

## Introduction

Peutz–Jeghers syndrome (PJS, OMIM 175200) is a rare autosomal dominant hereditary disorder characterized by mucocutaneous pigmentations and multiple gastrointestinal hamartomas. The incidence of PJS was estimated to be between 1:8300 and 1:200,000 births [1]. Studies have shown that PJS has an obvious familial aggregation tendency and *STK11* (serine/threonine protein kinase 11, OMIM 602216) located in the p13.3 region of chromosome 19, is the pathogenic gene of PJS [2, 3]. The germline mutation of *STK11* can be found in over 90% of patients who meet the clinical criteria of PJS [4].

As a high-risk group for malignant tumours [5], PJS patients have a significantly increased risk of gastrointestinal and extragastrointestinal malignancies [6], as well as high lifetime cumulative cancer risks. The risk of cancer is increased by 9.9 to 18 times for PJS patients compared with the general population [7]. Tumour sites are common in the rectum, stomach, and small intestine, followed by the breast and reproductive system, pancreas, and lungs [8]. In vitro studies have confirmed that overexpression of *STK11* in tumor cell lines can block tumour cells in G1 phase, thereby inhibiting tumour cell growth [9]. Therefore, patients with PJS may have a significantly higher risk of cancer due to *STK11* gene mutations.

Due to the familial aggregation of PJS, immediate family members may carry an *STK11* mutation and be in as much risk as the affected individual. Once the patient is clinically diagnosed or highly suspected of PJS, appropriate genetic counselling with subsequent genetic testing they should be provided. Similar genetic testing should also be targeted at those family members most likely to carry the pathogenic variants. Based on the clarification of the patient's family genetic background, tailored monitoring and management should be offered to all pathogenic mutation carriers to reduce the risk of polyp recurrence and malignancy. As a promising and effective method for PJS control, genetic testing of *STK11* for PJS is attracting increased attention from diverse specialists and has been incorporated into recent guidelines and consensus as the main genetic management measure to promote the early screening and diagnosis of PJS. However, due to the autosomal dominant inherited manner of PJS, there is still a 1/2 chance of the disorder being passed on to the patient's offspring [10]. Therefore, patients who have reproductive needs usually want to understand the risks of PJS for offspring and wish to prevent transmission to their offspring.

Preimplantation genetic testing for monogenic defects (PGT-M) is considered an ideal way to help PJS patients or at-risk people avoid transmitting the disease to offspring. It is a beneficial strategy for Mendelian disease using diverse genotyping methodologies such as array-based comparative genomic hybridization (aCGH), single nucleotide polymorphism (SNP) microarray, quantitative polymerase chain reaction (PCR), and next-generation sequencing (NGS). Currently, scientific management guiding the avoidance of PJS transmission through PGT-M remains sparse. This absence of guidelines is not conducive for physicians to comprehensively treat the patient or meet the reproductive needs of patients who want to have healthy mutation-free offspring. Thus, there is an urgent need to adopt comprehensive and effective guidelines including a responsible reproductive strategy for patients with reproductive intent while coordinating the treatment. However, as PJS is a multisystem disease that involves diverse medical disciplines, it is generally difficult for experts in a single field to assess the status of PJS patients from different perspectives and reasonably coordinate clinical treatment as well as assisted reproductive strategy. Based on the above, medical specialists with complementary expertise in the PJS field are required to work together to continuously improve and update the clinical guidelines of PJS.

In this study, we retrospectively analysed the clinical data of 51 PJS patients and developed a management flowchart recommendation specialized in prevention of PJS transmission. Under its guideline, a comprehensive PGT-M process by karyomapping to detect the mutation carrier status of the embryo was conducted on 4 PJS pedigrees. 2 healthy live births free of pathogenic mutation were obtained in 2 families, validating the feasibility and effectiveness of our strategy. Overall, this work made an important step forward towards the real clinical utility regarding PGT-M in the avoidance of PJS transmission.

## Methods

### Hospital-based clinical retrospective analysis

We retrospectively collected clinical the data of PJS patients who came to the First Affiliated Hospital of Zhengzhou University from January 2016 to January 2021 and analysed the sex, age at diagnosis, endoscopic characteristics, and outcomes of this patient group. Follow-up data were obtained from hospital records and telephone interviews with the patients or relatives. The start time of follow-up was defined as the time when the patient was diagnosed with PJS, and the end time of follow-up was defined as the death of the patient, the time of loss to follow-up, or the follow-up deadline 2021.03.02. This study was approved by the Ethics Committee of the First Affiliated University Hospital of Zhengzhou University.

### Assisted reproduction process through preimplantation genetic testing

#### Patients participating in PGT-M

Four PJS families were involved in the PGT-M process, including 4 PJS patients and their familial probands. These 4 patients were from 51 patients in the retrospective analysis who voluntarily underwent the PGT process. Four couples of PJS patients from different families received genetic counselling and assisted reproductive technology (ART) by PGT-M. Each couple consisted of a patient with PJS and their unaffected partner. This study was approved by the First Affiliated Hospital of Zhengzhou University, and all patients signed an informed consent form.

#### Gene mutation detection

Genomic DNA of the proband was extracted from peripheral blood through the QIAamp DNA Blood Mini Kit (Qiagen, Germany), and the extracted DNA was subjected to whole exome sequencing (WES), including library construction, probe capture, and next-generation sequencing (NGS). Sanger sequencing was used to verify the *STK11* gene mutation detected by NGS. The pathogenicity of mutations was evaluated according to ACMG genetic variation classification standards and guidelines and the ClinVar database (https://www.ncbi.nlm.nih.gov/clinvar/).

### Workflow of the karyomapping-based strategy

The workflow of the strategy is shown in Fig. 1a. First, TE cells from the embryo were lysed in lysis buffer to extract the DNA and then subjected to multiple displacement amplification (MDA). Second, the amplified DNA was applied to the karyomap SNP chip for further analysis. Subsequently, SNPs flanking the mutation were designed and haplotype analysis was carried out to identify the carrier status of the biopsied embryos. The CNV detection was also conducted to screen out aneuploidy. Finally, according to the comparison of haplotypes between the embryo and affected parents, probands. Euploid embryos without pathogenic mutations were deduced and transferred to the mother's uterus.

**Fig. 1:** PGT-M strategy for Peutz–Jeghers syndrome. **a** Workflow of PGT-M by karyomapping. **b** Pedigree diagram and linkage analysis identified for the disease-carrying allele. *M* Male, unaffected; *F* Female, affected; *R* Reference (proband), female’s brother; *E* Embryo. We sequenced the amplified genomes from each embryo, couple, and proband. This is the pedigree diagram of case 4 in the second PGT-M cycle. The SNPs within a range of 2 Mb upstream or downstream flanking the *STK11* gene are shown on the left. The heterozygous SNPs (AB) for the male and homozygous SNPs (AA or BB) for the female and female brothers were applied in the linkage analyses. Yellow bars indicate the pathogenic allele in the female’s brother inherited from the female to embryos E3, E4, and E7. **c** Results of CNV detection of embryos. Top left: CNVs of normal embryos E1, E2, E5, and E6 by karyomapping microarray. Top right: Abnormal E3 embryos with monosomy of the 22nd chromosome. Lower left: Abnormal E4 embryos with deletion of the 10th chromosome. Lower right: Abnormal E7 embryos with deletion of the 9th chromosome

### Embryo biopsy and single-cell whole genome amplification (WGA)

All the subject couples received assisted reproductive technology, using long GnRH agonist protocols for controlled ovulation. Then, the mature oocytes were fertilized by intracytoplasmic sperm injection, and the embryos were cultured in vitro according to the standard protocol. To obtain a sufficient amount of DNA fragments for subsequent analysis, a biopsy of the trophectoderm cells of embryos at the blastocyst stage (Day 5 or Day 6) was performed, subsequently, the biopsied 3–5 TE cells were placed in the EP tube containing PBS and WGA was carried out by multiple displacement amplification [11] (MDA). MDA followed the standard protocol provided by the QIAGEN REPLI-g Single Cell kit. The main steps were as follows: 4 µl of sample and 3 µl of buffer solution were mixed and incubated at 65 °C for 10 min, after which 3 µl of stop solution was added. Then, the total reaction system reached 50 µl by adding 40 µl MasterMix, followed by incubation at 30 °C for 8 h and storage at 4 °C after 3 min at 65 °C.

### Karyomap gene chip detection

Karyomapping gene chip detection was performed on the embryonic DNA samples after WGA and the peripheral blood samples of the subjects and couples. The specific steps were carried out according to the instructions of the Karyomap chip, including DNA fragmentation, precipitation, resuspension, hybridization, washing, extension, and colouring. Finally, the amplified DNA was scanned on the HumanKaryomap-12 Bead Chips (Illumina) platform, and the results were analysed by BlueFuse Multi (Illumina) software.

### Linkage analysis and aneuploidy detection

The *STK11* gene is located at 19p13.3. The range of 2 M upstream and downstream of the gene is selected as the main analysis area to determine the informative SNP. Informative SNPs are the main basis for judging which chromosome the embryo inherits from its parent. SNPs that can be used for linkage analysis need to meet the following conditions: (i). The proband's allele is a homozygous genotype at this locus. (ii). The allele of the PJS patient in parents was heterozygous, and the other was homozygous. Combining the SNP data of the proband’s genome NGS and the results of the linkage analysis of the karyomap chip, we constructed haplotypes related to the *STK11* mutation and inferred whether the embryo carries a chromosome containing the *STK11* mutation. Simultaneously, the original SNP data of the chip and BlueFuse Multi software (Illumina) were used to identify the whole-genome copy number variation (CNVs) of blastocysts. The results of the B-allele frequency and log R ratio charts were based on strict criteria to determine whether there was aneuploidy. At least two laboratory technicians reviewed all the steps.

### Frozen embryo transfer (FET) and prenatal diagnosis (PND)

Blastocysts with normal karyotypes and those that did not carry mutations were transferred back to the mother's uterus through FET. Amniotic fluid genetic testing at 18–22 weeks of gestation confirmed this result.

## Results

### Hospital-based clinical retrospective analysis

#### Basic clinical characteristics and family history

A total of 51 PJS patients admitted to the First Affiliated Hospital of Zhengzhou University were retrospectively enrolled, including 26 males and 25 females, with an average age of 29.2 years (7–65 years). The clinical characteristics of the patients are shown in Table 1. The average age of the first presentation of clinical symptoms was 17.9 years (1–54 years). The average age of the first diagnosis of PJS was 24.3 years (4–56 years). There were 21 cases with a clear family history of PJS, among which 8 cases had fathers suffering from the disease (including 1 sister with PJS); 7 cases had mothers suffering from the disease (including 3 brothers with PJS), the relatives of 3 patients are sons, and the relatives of 2 patients are daughters, respectively. In addition, 1 patient had a grandmother, mother, uncle, and sister suffering from the disease. These relatives were not included in the retrospective analysis.

**Table 1:** Baseline characteristics, fertility aspects, and follow-up outcome of 51 patients with Peutz–Jeghers syndrome

Demographics	Male	Female	Total
Number of patients	26	25	51
Mucocutaneous pigmentation, n (%)	16/26 (61.54%)	16/25 (64.00%)	32/51 (62.75%)
Age of presentation, years (mean ± SD)	17.9 ± 15.4	20.7 ± 13.9	19.2 ± 14.6
Age at diagnosis, years (mean ± SD)	24.3 ± 14.8	24.2 ± 14.1	24.3 ± 14.3
First clinical symptoms, n (%)			
Pigmentation	10/26 (38.46%)	7/25 (28.00%)	17/51 (33.33%)
Abdominal pain	6/26 (23.08%)	10/25 (40.00%)	16/51 (31.37%)
Hematochezia	3/26 (11.54%)	4/25 (16.00%)	7/51 (13.73%)
Location, n (%)			
Stomach	12/26 (46.15%)	7/25(28.00%)	19/40 (47.50%)
Colon	13/26 (50.00%)	9/25(36.00%)	22/40 (55.00%)
Rectum	5/26 (19..23%)	4/25(16.00%)	9/40 (22.50%)
Duodenum	6/26 (26.08%)	1/25 (4.00%)	7/40 (17.50%)
Polyp pathology, n (%)			
Hamartomatous polyps	12/26 (46,15%)	13/25 (52.00%)	25/51 (49.02%)
Inflammatory polyps	1/26 (3.85%)	3/25 (12.00%)	4/51 (7.84%)
Hyperplastic polyps	1/26 (3.85%)	2/25 (8.00%)	3/51 (5.88%)
Adenomatous polyp	1/26 (3.85%)	1/25 (4.00%)	2/51 (3.92%)
Adenocarcinoma	0	1/25 (4.00%)	1/51 (1.96%)
Recurrence rate of PJ polyp, n (%)	2/18 (11.76%)	1/17 (6.67%)	3/35 (9.38%)
Incidence of cancer,n (%)	3/18 (17.64%)	2/17 (13.33%)	5/35 (15.63%)
Mortality, n (%)	3/18 (17.64%)	1/17 (6.67%)	4/35 (12.50%)
Family history, n (%)	15/26 (57.69%)	6/25 (24.00%)	21/51 (41.18%)
Giving birth to affected offspring, n (%)	2/26 (7.69%)	3/25 (12%)	5/51 (9.8%)
Genetic testing performed, n (%)	2/26 (7.69%))	3/25 (12%)	5/51 (9.8%)
Fertility demand, n (%)	7/18 (30.77%)	6/17 (24.00%)	13/36 (25.49%)
Willing to perform PGT, n (%)	3/18 (11.15%)	4/17 (16.00%)	7/36 (13.73%)

### Clinical manifestations

Among the 51 patients, 32 had typical mucocutaneous pigmentation (62.75%), and 3 had solitary mucocutaneous pigmentation. Pigmentation on the lip or oral mucosa was found in all 32 cases, with 6 cases diagnosed with pigmentation on the extremities (fingertip, palm, etc.). The first clinical symptoms occurred during childhood or adolescence and included hyperpigmentation and gastrointestinal symptoms such as abdominal pain, abdominal cramps, hematochezia, and diarrhea. The diameter of pigmentation was generally 0.3–0.9 mm, irregular in shape, scattered, or densely distributed; other symptoms of PJS, as shown in our cases, were bellyache (16/51, 31.37%), hematochezia (7/51, 13.73%), and anal prolapse for 1 case (1/51, 1.96%). Some patients had gastrointestinal complications, such as intussusception in 3 cases and obstruction in 1 case.

### Endoscopy and imaging examination

The patients underwent gastrointestinal endoscopy and imaging evaluations. In 51 cases of PJS, 40 cases (78.43%) had gastrointestinal polyps, of which 35 cases had multiple polyps and 5 cases had 1–3 polyps. The gastrointestinal polyps of PJS are widely distributed, involving the stomach, duodenum, small intestine, colon, rectum, and other parts. According to endoscopic procedures, 19 cases (47.50%) of gastric polyps, 22 cases of colon polyps (55.00%), 9 (22.50%) cases of rectal polyps, 7 cases (17.50%) of duodenal polyps, 2 cases (5.00%) of small intestine polyps were detected, and there were 2 cases of polyps located in the ileocecal area (5.00%). Gastrointestinal polyps varied in the range between 0.3 and 5 cm in diameter, and were classified into pedicle and broad-based polyps, ranging from a few to hundreds. According to the literature, polyps may also occur outside the gastrointestinal tract, such as in the renal pelvis, urinary bladder, ureters, lungs, nares, and gallbladder which adds a certain degree of difficulty to the judgement and diagnosis of this disease. However, none of the 51 patients in this group had extragastrointestinal polyps.

### Histopathological results

Histopathological examination revealed the following results: 25 typical PJ hamartomatous polyps; 4 inflammatory polyps; 2 hyperplastic polyps, 2 villous tubular adenomas with local low-grade intraepithelial neoplasia; 2 gastric fundus gland polyps; 2 adenomatous polyps;1 gastric body polyp; 1 sessile serrated polyp; 1 tubular adenoma and 1 moderately differentiated adenocarcinoma.

### Genetic test results

Among 51 patients, a total of 5 voluntarily underwent genetic testing of PJS. The results showed that 5 patients all carried serine/threonine protein kinase (serine/threonine kinase 11, *STK11*) gene mutations, including *STK11* c.862+2T>G, *STK11*c.911G>C, *STK11*c.527A>G, *STK11*c.580G>A, *STK11*EX1DEL and EX8-9DEL. The genetic test results of 4 cases involved in the PGT-M process are shown in Table 2. The remaining 1 case was a proband that underwent *STK11* gene mutation detection (whole-exome sequencing and MLPA). The results showed that this patient had a heterozygous mutation in STK11(*STK11*:NM_000455: c.862+2T>G), which might affect mRNA splicing and protein function. According to the guidelines of the American Society of Medical Genetics and Genomes (ACMG), the mutation was a likely pathogenic mutation, and not found in his parents as the genetic test indicated.

**Table 2:** Characteristics of the couples involved in PGT-M

Patient ID	Patient gender	Female age	Female karyotype	Male age	Male karyotype	Mutation assessed	Reference source	ACMG	ClinVar	Cycle	No. of retrieved oocytes	No. of MII oocytes	No. of biopsied blastocysts
Case1	Male	27	46,XX	30	46,XY	*STK11*c.911G>C (p.Arg304Pro)	Husband's father	P	P	1	13	12	5
Case2	Male	36	46,XX	36	46,XY	*STK11*c.527A>G (p.D176G)	Couple's daughter	LP	LP	1	6	6	4
Case3	Female	28	46,XX	28	46,XY	*STK11*c.580G>A (P.Asp194.Asn)	Husband's father	P	P/LP	1	24	20	13
Case4	Female	30	46,XX	28	46,XY	*STK11*EX1DEL and EX8-9DEL	Wife's brother	P	–	1	22	21	3
Case4	Female	30	46,XX	28	46,XY	*STK11*EX1DEL and EX8-9DEL	Wife's brother	P	–	2	23	22	7

*ACMG* American College of Medical Genetics, *LP *likely pathogenic, *P* pathogenic

### Treatment methods

A total of 76.47% (39/51) of PJS patients underwent endoscopic therapy, of whom 84.62% (33/39) underwent endoscopic polypectomy or electrocoagulation, and 5.13% (2/39) received argon plasma coagulation (APC), similar to endoscopic polypectomy accompanied by APC (2/39). Only 2 patients received endoscopic mucosal resection (EMR), and endoscopic submucosal dissection (ESD). Seventeen patients underwent surgical operations including 88.24% (15/17) who received surgical intervention for removal of the polyps. Due to a complicated condition, the remaining 1 patient underwent intestinal adhesion lysis, ascending colon and jejunum multiple polyp extraction, and small intestinal intussusception manual reduction. Another patient underwent intussusception reduction and resection of multiple polyps in the large and small intestines.

### Fertility aspects of PJS patients

In all 51 patients, 5 (9.8%) showed that PJS had affected their children. Of the 36 respondents, 13 (25.49%, mean age 32 years) indicated reproductive intent despite PJS. Meanwhile, 7 (13.73%) reported that PGT technology influenced their attitude to have children and would consider the PGT process. Finally, 4 (13.73%) patients decided to participate in the PGT-M process.

### Follow-up and prognosis

Of the 51 cases, 36 completed the follow-up for 6 months to 15 years, and 15 refused or were lost to follow-up. One of the patients lost to follow-up had pancreatic cancer, and the current condition is unknown. In our report of 36 patients who completed the follow-up, 27 patients showed stable conditions, while some of them had intermittent abdominal pain. Among the remaining 9 cases, 2 females and 1 male encountered polyp recurrence after 5 years of surgical treatment. The prognosis of these 3 patients was as follows:1 female died of cachexia caused by ovarian malignant transformation and intestinal obstruction, another female patient is currently being treated in another hospital and the male died of colon cancer due to rapid disease progression. In addition to the above cases, there were also 2 male patients who died; unfortunately, the reasons were unknown due to the family members' refusal to follow up. One patient with rectal cancer and 1 patient with colon cancer recovered well after radical surgery, 1 patient with ovarian cancer was waiting for elective surgical treatment, and 1 patient had a postoperative intestinal fistula.

### PGT-M results

#### Mutation detection

According to ACMG, four Pathogenic (P) or Likely Pathogenic (LP) *STK11* gene mutations were detected in 4 families (case 1: *STK11*c.911G>C, p.Arg304Pro; case2: *STK11*c.527A>G, p.D176G; case3: *STK11* c.580G>A, P.Asp194.Asn; case4: *STK11*EX1DEL and EX8-9DEL). All mutations were confirmed by the Sanger sequencing results of the proband.

#### Single-cell whole genome amplification

Single-cell WGA and aneuploidy detection were performed on 32 blastocysts of 4 couples from 5 PGT-M cycles, among which case 4 was carried out for two cycles, and the average number of blastocyst biopsies per PGT-M cycle was 6.4. Trophoblast cell (TE cell) were used for WGA using the MDA method, and the DNA of all embryonic TE cells was successfully amplified (32/32).

#### Determination of informative SNP

The *STK11* gene is located in the 13p21.32-p21.33 segment of chromosome 19. The start and stop positions are 1189406 and 1228248, respectively, and the size of the region is approximately 39 kb. We determined the main analysis zone of *STK11* at the region 189406–2228248, and the analysis size was approximately 2.0 Mb. In addition, the 5' upstream and 3' ends of the region were selected as auxiliary analysis areas. SNP information of each case is shown in Table 3 and Additional file 1: Table S1-4.

**Table 3:** Informative SNPs flanking *STK11*gene of Peutz–Jeghers syndrome in case4

Red font indicates SNPs associated with pathogenic mutation

#### Haplotype analysis of *STK11* gene by karyomap microarray

The karyomap chip was used to perform genotype analysis of SNP alleles at SNP sites designed within the 2 M range upstream and downstream of the *STK11* gene. According to the genotype of the proband, the haplotype linked to the *STK11* mutant allele was identified. The results indicated that haplotypes associated with *STK11* mutant alleles were found in 5 cycles of 4 couples. The number of informational SNPs used to establish haplotypes is 7, 36, 20, 8, and 8.

Taking the second cycle of case 4 as an example, there were a total of 8 available SNPs (see Table 3). The mother and her brother were diagnosed with PJS and the STK11 gene mutation was detected in both of them, therefore the mother's brother was determined as a reference. When we judged whether E1 carried the mutation, we first checked the locus rs1108114 and showed that the brother was A/A, the mother was A/B, the father was A/A, embryo 1 was A/B, and both the mother and her brother had the A allele. Thus, it could be inferred that allele A of the mother and brother was pathogenic and that allele B of the mother was nonpathogenic. Meanwhile, the homozygous A/A father could only transmit allele A to E1, which meant that E1 (A/B) inherited the mother's nonpathogenic allele B. In summary, both alleles of E1 (A/B) were nonpathogenic. Other SNPs could also be inferred by the same method. Finally, the haplotypes of all the embryos inherited from the mother were deduced to determine whether the embryo was an *STK11* mutation carrier. The haplotype results are shown in Fig. 1b. Among the 7 blastocysts tested, embryos 3, 4, and 7 were maternal mutation carriers, and the rest were nonmaternal mutation carriers.

#### Embryo selection of non *STK11* mutation carriers and results of frozen embryo transfer

Based on embryo aneuploidy and linkage analysis, a total of 15 embryos were identified as normal and transferable embryos. The average number of embryos that can be transferred per PGT-M cycle was 3 (specific results are shown in Table 4). Two couples (cases 2 and 3) underwent frozen embryo transfer (FET) and clinical pregnancy. Unfortunately, the transferred embryos of case 1 and case 4 did not achieve clinical pregnancy. Thereafter, amniotic fluid samples obtained at 20 weeks were collected from women who were successfully clinically pregnant for foetal karyotyping and the results of PGT-M were confirmed by detecting the *STK11* gene mutation of gDNA in amniotic cells. Two healthy live births were born in case 2 and case 3, and the remaining two embryos in case 4 were waiting transferration.

**Table 4:** The results of karyomapping analysis of embryos

Patient ID	Cycle	Embryo ID	Embryo days	CNV	Carrierstatus	Recommendation	Clinicaloutcomes
1	1	1	6	46,XX	Paternal mutation carrier	Not transferred	Abandoned
	1	2	6	46,XX	Normal homozygote	Transferred	No pregnancy
	1	3	6	46,XY,dup(3) (q29 → q24)	Paternal mutation carrier	Not transferred	Abandoned
	1	4	6	46,XX	Paternal mutation carrier	Not transferred	Abandoned
	1	5	6	45,XY,-1	Normal homozygote	Not transferred	Abandoned
2	1	1	5	46,XY	Paternal mutation carrier	Not transferred	Abandoned
	1	2	5	46,XX	Normal homozygote	Transferred	Live birth
	1	3	5	46,XX	Normal homozygote	Transferred	Abandoned
	1	4	6	46,XX	Paternal mutation carrier	Not transferred	Abandoned
3	1	1	5	46,XX	Normal homozygote	Transferred	Live birth
	1	2	5	46,XX	Normal homozygote	Transferred	Abandoned
	1	3	5	46,XY	Maternal mutation carrier	Not transferred	Abandoned
	1	4	5	46,XY	Maternal mutation carrier	Not transferred	Abandoned
	1	5	5	46,XX	Normal homozygote	Transferred	Abandoned
	1	6	5	46,XX	Normal homozygote	Transferred	Abandoned
	1	7	5	46,XX	Maternal mutation carrier	Not transferred	Abandoned
	1	8	5	46,XX	Normal homozygote	Transferred	Abandoned
	1	9	6	46,XX	Normal homozygote	Transferred	Abandoned
	1	10	6	46,XY	Maternal mutation carrier	Not transferred	Abandoned
	1	11	6	46,XY	Normal homozygote	Transferred	Abandoned
	1	12	6	46,XY	Maternal mutation carrier	Not transferred	Abandoned
	1	13	6	46,XX	Maternal mutation carrier	Not transferred	Abandoned
4	1	1	5	46,XX	Maternal mutation carrier	Not transferred	Abandoned
	1	2	5	46,XX	Maternal mutation carrier	Not transferred	Abandoned
	1	3	6	46,XY	Normal homozygote	Transferred	No pregnancy
	2	1	5	46,XY	Normal homozygote	Transferred	No pregnancy
	2	2	6	46,XY	Normal homozygote	Transferred	No pregnancy
	2	3	6	45,XY,-22	Maternal mutation carrier	Not transferred	Abandoned
	2	4	6	46,XY,del(10) (q23.1-q26.3)	Maternal mutation carrier	Not transferred	Abandoned
	2	5	6	46,XX	Normal homozygote	Transferred	Cryopreservation
	2	6	6	46,XX	Normal homozygote	Transferred	Cryopreservation
	2	7	6	46,XX,del(9) (q31.1-qter)	Maternal mutation carrier	Not transferred	Abandoned

#### Aneuploidy detection

The results of the aneuploidy test showed that the euploidy ratio was 6.25% (2/32), and the chromosome abnormality ratio was 15.6% (5/32). In the 5 PGT-M stimulation cycles, the chromosomes of the embryos in the first cycle of case 2, 3, and case4 were all normal, and there were 5 embryos with abnormal chromosomes in the second cycle of case 1 and case 4 (see Fig. 1c, Table 3).

#### PJS genetics and gastrointestinal management flowchart

The management of PJS requires multidisciplinary specialist knowledge provided by diverse medical centres, such as the Gastroenterology Department and Reproductive Center, Department of Medical Genetics, and prenatal diagnosis. Therefore, a set of MDT (multidisciplinary treatment) based management recommendations for PJS patients were proposed (Fig. 2). An integral multidisciplinary team should include reproductive doctors, genetic specialists, gastroenterologists, surgeons, oncologists, physicians, pathologists, radiologists, and the nursing team. Gastroenterologists, surgeons, and physicians are responsible for the diagnosis, condition evaluation, and surgical planning. Pathologists and radiologists help analyse and explain the imaging and pathological results. Geneticists should participate in explaining the results of genetic testing and formulating the tailored PGD plan when the patients have reproductive needs. Reproductive doctors make the IVF-PGT plans, and oncologists are responsible for assessing the risk of tumours and guiding surveillance monitoring. If PJS patients are children, the MDT team should also involve paediatricians in developing a comprehensive treatment plan and individual evaluation.

**Fig. 2:** Flowchart of surveillance management of Peutz–Jeghers syndrome. *PJS* Peutz–Jeghers syndrome. Multidisciplinary MDT treatments included gastroenterology, surgical, oncology, imaging, and reproductive medicine. *GI:* Gastrointestinal; *PGT-M*: Preimplantation genetic testing for monogenetic defects. Pancreatic cancer and extra-GI cancer monitoring*: Extra-GI cancer should include breast, ovary, uterus, cervix, and testes cancers. Lung cancer can also be screened through chest CT or chest radiograph if the patient smokes. For all these cancers. Age to begin surveillance, surveillance interval and surveillance procedures should depend on local and MDT expertise

The main process of MDT shall follow these steps: First, clinically confirmed patients should undergo routine endoscopy and imaging examinations, and genetic testing is also recommended to all patients as one of the initial investigational examinations. Thereafter, the patient's attending physician should summarize the examination results and report them to the multidisciplinary team. Through the MDT process, specialists from related departments should comprehensively evaluate the patient's condition and reach a consensus to propose comprehensive plans for the patient, including the clinical management strategy, surgical treatment plan, and postoperative monitoring plan. Simultaneously, genetic counselling on reproductive risk and preimplantation genetic testing or prenatal diagnosis are recommended for patients with reproductive needs. Each specific plan should be continuously adjusted according to the dynamic changes of the patient's physical condition. The surveillance plans referred to the most recent gastrointestinal management of PJS endorsed by the European Society of Gastrointestinal Endoscopy (ESGE) and European Society for Paediatric Gastroenterology Hepatology and Nutrition (ESPGHAN) in 2019 [12, 13], Guidelines for the management of hereditary colorectal cancer from the British Society of Gastroenterology (BSG)/Association of Coloproctology of Great Britain and Ireland (ACPGBI)/United Kingdom Cancer Genetics Group (UKCGG)[14] and Genetic Testing and Management of Hereditary Gastrointestinal Cancer Syndromes by the American College of Gastroenterology(ACG) [15].

All PGT-M strategies were performed according to the ESHRE PGT Consortium good practice recommendations for the organization of PGT [16].

## Discussion

PJS is a rare autosomal dominant hereditary disease. Despite its low incidence and easy diagnosis, patients usually have severe clinical symptoms, as well as an elevated risk of cancer. Even if endoscopic or surgical treatment is performed, multiple polyps are still difficult to cure and complicated by diverse gastrointestinal complications. In addition, PJS may be inherited through a single dominant pleiotropic gene, with a high penetrance rate [17]. Both men and women can carry the pathogenic gene, and it is not uncommon to observe several people’s morbidity in a family. It not only harms patients’ health but also poses a serious threat to future generations. Therefore, prevention of the vertical transmission of pathogenic mutations to offspring is as important to patients as early diagnosis and treatment to some degree.

Based on our retrospective study of PJS patients in the Chinese population, we identified 51 individuals of which 4 were deceased. In general, the main characteristics of PJS are multiple gastrointestinal polyps, as well as pigmentation of the skin or mucous membrane which often appear at birth or in infancy. Our study showed that 62.75% (32/51) had oral mucosal pigmentation and 11.76% (6/51) had pigmented spots on the extremities. GI symptoms accounted for most of the first clinical symptoms (31/51 60.78%) which indicated that they were likely to be found as the first symptom preceding mucocutaneous pigmentations. This finding was in agreement with other reports that demonstrated gastrointestinal symptoms were the most common initial presentation [18, 19]. However, oral mucosal pigmentations should not be ignored since pigmentations are easier to assist physicians in the diagnosis by their noticeable PJS characteristics.

Among the 51 patients, the colon was the most affected segment, followed by the stomach, rectum, duodenum, small intestine, and ileocecal part. PJ polyps were found in the transverse or sigmoid colon in 43.14% of patients. According to the WHO Classification of Tumours of the Digestive System, the small intestine is the most common site of PJPs [20]. However, our study revealed only 7.84% of small intestinal polyps, while there was a higher incidence rate of colonic polyps and gastric polyps, and the reasons may be as follows: (i). The lower proportion of small intestinal endoscopy is due to the differences between China and Western countries in the selection of endoscopy. This may be related to widely applied gastroscopy and colonoscopy and the limited application of small intestinal endoscopy in Chinese patients, which may lead to a missed diagnosis. (ii). Due to economic reasons, some patients do not seek medical treatment until they have severe intolerable symptoms. As colonic polyps and gastric polyps reflected more severe symptoms than small intestinal polyps, they had an elevated detection rate.

At present, PJS treatment mainly includes endoscopic polyp resection and surgical operation. According to our study, the most common ones were resection or electrocoagulation of strangler (34 / 39, 87.18%), while APC, EMR, or ESD alone were rarely used. Moreover, as PJPs are usually small, sessile, multiple, and difficult to remove, patients always need multiple endoscopic treatments. The average number of endoscopic treatments in our study was approximately 2.5. Meanwhile, of the 51 patients, 17 patients mainly underwent surgical resection of polyps, among whom 2 patients were treated with polypectomy and relieved of complications after surgery.

PJS patients are a typical high-risk population for malignant tumours. The lesions inside and outside the digestive tract of PJs patients are prone to malignant transformation. Pancreatic cancer and breast cancer are the most common malignant tumours in PJS [21]. Our follow-up study found that the incidence of PJS combined with malignant tumours was 11.76% (6/51). Male patients mainly had involvement of the colon, rectum, and pancreas, and female patients mainly had involvement of the ovary. At present, the mechanism of malignant transformation in PJS patients is still controversial and needs further study. Because polyps can continue to grow after resection and have the tendency of canceration, regular re-examination and dynamic follow-up are needed. If possible, gene testing is recommended to guide further diagnosis, treatment and follow-up. Because PJS is hereditary in the family, the offspring of the patient should also be closely followed, and regular gastroscopy, enterobarium contrast, capsule endoscopy, and other examinations should be performed to avoid missed diagnosis or misdiagnosis. If the black spots of skin and mucous membrane are found in children or adolescents, we should ask family members if they have a similar medical history and further check the digestive tract to make a clear diagnosis as soon as possible and conduct minimally invasive endoscopic treatment in time to prevent the occurrence of acute intussusception or even canceration.

Regarding fertility aspects, our study demonstrated that approximately one-third of respondents had certain reproductive intent. Moreover, PGT influenced decisions regarding fertility planning in one-sixth of respondents who were willing to perform the PGT process. The majority of these patients underwent genetic testing, and finally, 4 patients participated in the PGT process. PGT was considered an efficient option to prevent the transmission of PJS to the next generation. Similarly, life questionnaire research on PJS patients showed that 40% of them changed reproductive life choices due to PJS [22]. Therefore, these results highlighted not only the timely clinical treatment for PJS patients but also that genetic counselling and subsequent PGT planning should be discussed by specialists.

Currently, with the advancement of PDG technology and the increasing reproductive demand for healthy offspring, guidelines of PJS regarding genetic aspects remain insufficient and it is often difficult to address the reproductive needs of patients. In our management flowchart, genetic management was formulated as an extremely important branch. Through the process of genetic counselling—mutation detection—risk assessment—PGT and ART- PND verification, patients will have a higher probability of obtaining healthy offspring. Meanwhile, the introduction of the MDT model to coordinate GI and genetic management can simultaneously complete the treatment and inherit transmission of PJS within a certain period to meet the health and reproductive needs of patients. Genetic risk assessment can also benefit patients or at-risk relatives and their offspring in the same pedigree. Finally, the highly personalized and dynamic surveillance plan created by the multidisciplinary team will take into account the patient’s gastrointestinal monitoring, tumour risk monitoring, and offspring genetic risk to minimize the risk of malignancy and recurrence of GI polyps.

Furthermore, through linkage analysis and aneuploidy detection following TE cell biopsy, we successfully screened 32 embryos from 4 PJS families. Healthy embryos proven to be free of chromosomal disorder without *STK11* mutation were transferred back to the mother through FET. Finally, two live births were born in the two families. The take-baby home rate was approximately 40%, which is slightly higher than that of the normal IVF cycle (33%) [23]. We believe that with the continuous improvement of PJS clinical management and the implementation of multidisciplinary treatment, a more targeted ART program tailored to patients will enable the clinical pregnancy rate of PJS patients to reach a more ideal level.

As the key method of PGT-M of PJS patients in this study, the strategy based on linkage analysis is an efficient and ideal method, which does not rely on high-throughput sequencing and has great application potential in PGT and PGS of monogenic diseases. This strategy will be described in more detail in the following sections, and we will discuss its advantages:

(i) High accuracy and reliability. Traditional PCR technology of DNA sequencing may cause low accuracy due to allele drop out (ADO), while Karyomap analyses the DNA amplification products of single or several cells, and combines several closely matched SNPs in the disease-causing gene region into a haplotype, followed by further analysis to distinguish the chromosomal region where the disease-causing gene is located from the normal chromosome region. This method is based on SNP genotyping technology and utilizes indirect analysis of linked polymorphisms, thus obtaining higher confidence than traditional single-cell PCR which is usually complicated with DNA contamination and an approximately 10% ADO rate [24]. In this report, all 32 embryos obtained ideal amplification and analysis results, which showed that the results of PGS using the Karyomap gene chip were reliable.
(ii) Low demands on patients. Depending only on the DNA of affected couples and probands, informative SNPs across each chromosome could be identified to construct parental haplotypes; thereafter, the haplotype inherence could be mapped to detect the positions of any crossovers in the proband as well as in the preimplantation embryos [25].
(iii) High efficiency. As long as a clear pathogenic region can be provided, PGT can be carried out with no patient-specific test, which greatly shortens the wait time, saves resources, and reduces the anxiety of patients. The whole experimental process can be completed within 5 days, meeting the needs of most laboratories and patients.
(iv) Aneuploid screening PGS can be performed simultaneously. As a kind of SNP chip, a karyomap gene chip can not only perform PGS but also distinguish chromatid and trisomy better than traditional microarray-based comparative genomic hybridization (array CGH) technology. The principle is that SNP genotyping and genotype interpretation help to distinguish monosomic, trisomic, and single parent diploids that array CGHs cannot distinguish.
(v) Reduced damage caused by unnecessary interventions. Compared with prenatal diagnosis, the effective screening of embryos using karyomapping linkage analysis and aneuploidy detection improves the probability of healthy nonmutated foetuses obtaining clinical pregnancy (the no-carrier mutation rate is above 90%) and largely avoids the risks of multiple induced labourers caused by the potential failure of prenatal diagnosis to the female reproductive system and psychology.

However, this strategy still has limitations. First, linkage analysis is needed based on the results of haplotype analysis, in which clear pedigree information and probands are necessary. In addition, it cannot detect novel mutations or duplication of equivalent sequences. Therefore, the application of karyomapping technology is limited to monogenetic diseases with a definitive genetic diagnosis and well-established pedigree conditions. Second, haplotype analysis of the karyomapping strategy is different from direct sequencing. The possible recombination within alleles increases the uncertainty of the analysis results, since the occurrence of recombination may lead to base or sequence changes between adjacent SNP loci for haplotype analysis, and then impair the accuracy of linkage analysis. However, recombination within alleles is indicated to have a low probability, as recombination is regulated by a very conservative mechanism and does not occur randomly [26]. Through prenatal diagnosis technology of amniocentesis at 20 weeks of gestation, we can avoid missed diagnosis and misdiagnosis caused by recombination to the greatest extent.

In conclusion, we summarize the clinical and genetic aspects of PJS as well as the management flowchart of this rare cancer predisposition syndrome, highlighting the need for a multidisciplinary approach containing genetic management and the creation of prospective and consensus guidelines on multidisciplines in the future. Furthermore, we report a feasible and efficient PGT-M strategy to increase the identification of embryo pathogenic mutation carrier status and confirm its feasibility and effectiveness. Avoidance of PJS transmission to offspring of patients and families who would benefit from this method is critical in improving the quality of life of these patient groups. In the upcoming era of massively parallel sequencing being used for clinical genetic testing, whole-exome sequencing and even whole-genome sequencing will be considered for the clinical management of PJS to identify pathogenic variants and single-nucleotide polymorphisms. More importantly, when PJS is diagnosed, a multidisciplinary team including genetic specialists, gastroenterologists, surgeons, oncologists, physicians, and the nursing team should evaluate the prognosis of the disease and provide efficient management and surveillance programs.

### Supplementary Information

**Additional file 1: Table S1.** Informative SNPs flanking STK11gene of Peutz–Jeghers syndrome in case1

## Data Availability

The data that support the results of this study can be obtained from the corresponding author, upon reasonable request.

## Abbreviations

PJS: Peutz Jeghers syndrome
PGT-M: Preimplantation genetic testing for monogenic defects
MDT: Multidisciplinary team
ART: Assisted reproductive technology
FET: Frozen embryo transfer
PND: Prenatal diagnosis
MDA: Multiple displacement amplification
WGA: Whole genome amplification
TE: Trophectoderm
